# Exosomal miRNAs in hepatitis B virus related liver disease: a new hope for biomarker

**DOI:** 10.1186/s13099-020-00353-w

**Published:** 2020-04-24

**Authors:** Manikankana Bandopadhyay, Mausumi Bharadwaj

**Affiliations:** Molecular Genetics and Biochemistry, National Institute of Cancer Prevention and Research (NICPR), Indian Council of Medical Research (ICMR), Noida, Uttar Pradesh 201301 India

**Keywords:** Hepatitis B virus, miRNA, Exosome, Hepatocellular carcinoma

## Abstract

The World Health Organisation, in its 2019 progress report on HIV, viral hepatitis and STDs indicates that 257 million people are afflicted with chronic HBV infections, of which, 1 million patients lose their lives every year due to HBV related chronic liver diseases including serious complications such as liver cirrhosis and hepatocellular carcinoma. The course of HBV infection and associated liver injury depend on several host factors, genetic variability of the virus, and the host viral interplay. The challenge of medical science is the early diagnosis/identification of the potential for development of fatal complications like liver cirrhosis and HCC so that timely medical intervention can improve the chances of survival. Currently, neither the vaccination regime nor the diagnostic methods are completely effective as reflected in the high number of annual deaths. It is evident from numerous publications that microRNAs (miRNAs) are the critical regulators of gene expression and various cellular processes like proliferation, development, differentiation, apoptosis and tumorigenesis. Expressions of these diminutive RNAs are significantly affected in cancerous tissues as a result of numerous genomic and epigenetic modifications. Exosomes are membrane-derived vesicles (30–100 nm) secreted by normal as well as malignant cells, and are present in all body fluids. They are recognized as critical molecules in intercellular communication between cells through horizontal transfer of information via their cargo, which includes selective proteins, mRNAs and miRNAs. Exosomal miRNAs are transferred to recipient cells where they can regulate target gene expression. This provides an insight into the elementary biology of cancer progression and therefore the development of therapeutic approaches. This concise review outlines various on-going research on miRNA mediated regulation of HBV pathogenesis with special emphasis on association of exosomal miRNA in advanced stage liver disease like hepatocellular carcinoma. This review also discusses the possible use of exosomal miRNAs as biomarkers in the early detection of HCC and liver cirrhosis.

## Background

Globally, 247 million people are affected with chronic Hepatitis B virus (HBV) infection [1]. Although there is availability of operative vaccine for HBV, but cost and non-responsiveness of vaccine added to vaccine escape mutant viruses continue to identify HBV infection as a major global health concern [2–5]. HBV is one of the important human DNA viruses that belong to the Hepadnaviridae family [6]. It is hepatotropic non-cytopath-ic virus having strong oncogenic potential [7]. HBV is often associated with acute and chronic infections of the liver and chronic HBV infections in turn can lead to severe liver complications like developing advanced liver diseases such as liver cirrhosis (LC) and hepa-tocellular carcinoma (HCC).

Liver cirrhosis is the 11th most common cause of death worldwide and is a growing cause of morbidity and mortality in developed countries [8, 9]. Though HBV and HCV infection, alcohol intake and non-alcoholic liver diseases are the main causes of liver cirrhosis in developed countries, HBV infection is the most common cause of liver cirrhosis in sub-Saharan Africa and most parts of Asia [10]. The occurrence of Hepatocellular carcinoma (HCC) is the sixth highest amongst all cancers and is the third most common cause of cancer-related deaths in the world. High recurrence and metastasis rates have become the major impediment to improve long-term survival of HCC patients [11, 12].

Exosomes are emanating as key mediators of intercellular communication, since they carry nucleic acids, proteins and lipids that can be transported to a recipient cell. Exosomes are small vesicles (30–100 nm) secreted by many cells. Exosomes derive from early endosomes that fuse with multi-vesicular bodies from where individual vesicles (exosomes) are released in the extracellular space. Bio-fluids like plasma/serum, urine, breast milk, and cerebrospinal fluid (CSF) are the potential carrier of exosomes [13, 14]. The exosomes contain a lipid bilayer which is known to encapsulate proteins, selected miRNAs and mRNAs and protects them from degradation. Exosomal proteins, mRNAs, and miRNAs are therefore functionally active [15, 16]. Since exosome contains selective miRNA that differ from the cell of origin, these secreted vesicles may play an important role in normal physiological processes and also may be exploited in conditions like viral infections. Some exosomes function as pro-tumorigenic factors that can mediate intercellular communication in the tumor microenvironment via exosomal miRNA which contribute to cancer progression. This review highlights the findings regarding the involvement of miRNA in various aspect of hepatitis B biology and potential role of exosome derived miRNAs as a means of intercellular communication in end stage liver disease such as hepatic cancer.

## Exosomes

There are at least three extracellular vesicles (EVs) in the extracellular microenvironment, classified as exosomes, micro vesicles (MVs) and apoptotic bodies (ABs) according to their size and mechanism of formation. Though both MV and exosomes comprise proteins and nucleic acids, they differ in size, with MVs ranging from 100 to 1000 nm while exosomes are approximately 100 nm in diameter. ABs are released from the apoptotic cells, and contain fragmented nuclei and intracellular organelle. AB measures approximately 1 μm or more in diameter. Although AB and MV are directly formed and released by the cell membrane, exosomes are secreted through the process of endocytosis of the multivesicular bodies (MVBs) [17]. Differentiation can be made amongst the three EVs on the basis of the RNA contained in them. ABs predominantly contain ribosomal RNA (rRNA), whereas MVs contain virtually no RNA. Exosomes are characterized by large amounts of low molecular weight RNA but carry no rRNA. Further, each vesicle also differs in the surface molecules expressed, such as phosphatidylserine on ABs; integrin, secretin and CD40 on MVs, and tetraspanins on exosomes [18]. Exosomes, a subset of extracellular vesicles, are known to function as intercellular communication vehicles as they carry components such as DNA, mRNA, miRNA, proteins, lipids and transcriptional factors. The transfer of molecular pathogenic contents facilitates long-distance crosstalk between cancer cells and distant organs, thereby engendering preliminary steps for pre-metastatic niche formation.

### Historical standpoint, biogenesis and composition

The term exosome is first used by Trams et al. in the early 1980s [19]. It was believed that during red blood cell maturation, the transferrin receptor and many membrane-associated proteins were shed in small membrane vesicles by an unidentified secretory process [20, 21]. This process was considered as a cellular approach to discard unwanted proteins and molecules, with exosomes functioning as cellular waste disposals.

Exosomes do not originate by direct budding or shedding of plasma membrane [22]. They are formed via inward budding of endosomal membranes, thereby resulting in the formation of intracellular multivesicular bodies (MVB). The latter fuse with plasma membrane and release exosomes to the exterior [23, 24].

The exosomes contain a lipid bilayer which is known to encapsulate proteins, selected miRNAs and mRNAs and protects them from degradation thereby retaining the functional activity of the components. Recent investigations have revealed the presence of long non-coding RNAs (lncRNAs) in exosomes and these could potentially act as biomarkers for occurrence of cancer [25, 26]. Exosomes also contain genetic materials of viruses/prions. Exosomes secreted from hepatitis C virus (HCV) infected cells contain full-length viral RNA and protein. These exosomes are capable of transmitting infection to other hepatocytes [27, 28]. Exosomes isolated from the sera of chronic HCV-infected patients contain HCV RNA. These exosomes could facilitate viral receptor-independent transmission of HCV to hepatocytes [29]. All exosomes share common proteins/protein families that could serve as exosomal markers. These proteins consist of membrane-associated proteins, such as tetraspanin CD9, CD63, CD81, CD82; cytoplasmic proteins, such as Hsp 70 and Hsp90; transport associated protein Alix and TSG101; and membrane transport and fusion proteins, such as Rab GTPases and annexins [22, 30–32].

### Isolation and function

Due to their small size and low density, exosome isolation regularly involves multiple centrifugation and ultracentrifugation steps with a rotational force up to 100,000 × g for sedimentation. Sometimes, centrifugation is also combined with 0.1 μm to 0.22 μm filtration in order to separate the nano-sized particles and to eliminate larger particles and cellular debris [33]. Immunoaffinity capture methods can be used as a way to circumvent any ultracentrifugation process to isolate exosomes from cancer cells or patient serum samples using beads coated with antibodies against any exosome-specific surface marker, such as the tetraspanins, CD63 or CD82.

There are multiple ways by which cells interact with each other like direct membrane-to-membrane connection or secretion of soluble mediators. Currently exosomes have appeared as important mediators of cellular communication. The main function of exosomes is to participate in cell-to-cell communication by transporting bioactive molecules to recipient cells near to or distant from the original cells. Additionally, they are involved in normal physiological processes, like lactation, immune reaction, neurological function, and development and advancement of disease, for example, liver disease [34], neurodegenerative diseases, and cancer [35]. Diverse types of hepatitis viruses, such as HBV, HCV utilize exosomes to transfer signalling-competent proteins and functional microRNAs to uninfected cells [36–38]. Exosomes may be a natural vehicle for the somatic to germ line transport of RNA [39]. Exosomes are closely related to tumor development, pre metastatic niche formation and metastasis [reviewed in [40] ]. Since the focus of this review paper is on exosomal miRNA in HBV related liver disease we shall concentrate our discussion towards various effects of exosomal miRNA (ignoring its other cellular components) on diverse biological functions.

## miRNAs

MicroRNAs (miRNAs) have emerged as a prominent tool to regulate gene expression through the RNA interference pathway. They are 19–23 nucleotides long, highly conserved, endogenous, small noncoding RNAs. Residues 2–8 of the miRNA are the most conserved among homologous metazoan miRNAs [41, 42]. Watson–Crick base pairing between the 3′-untranslated region (UTR) of the mRNA target and the 5′-end of miRNAs, particularly the ‘miRNA seed sequence’ (comprising of nucleotides 2–7), is an important determinant of functional target sites [43]. Based on the 2–7 nucleotide seed sequence match, single miRNA can bind and control multiple mRNAs function. On the other hand, a single mRNA can be targeted by multiple miRNAs. If there is incomplete matching between the miRNA and target mRNA, it will bring about the repression of translation, else, if there is a perfect match, it leads to the degradation of the target mRNA [43]. Mature miRNA incorporated as single-stranded RNA into a ribonucleoprotein complex known as the RNA-induced silencing complex (RISC). The RISC recognizes target gene sequences based on perfect (or nearly perfect) complementarity between the miRNA and the mRNA. Next the endonuclease of the RISC cleaves the mRNA at a site near the middle of the miRNA complementarity, measuring from the 5′ end of the miRNA and cuts between the matching section of nucleotides 10 and 11 of the miRNA. Once mRNA is cleaved, the miRNA is released undamaged and can recognize and destroy the sequence of new mRNA. Two possibilities were put forward to explain the translational repression. After translation initiation though the density of the ribosomes on the message remains unaltered, but the slowing or stalling of all the ribosomes occurs on the message. An alternate possibility is that translation continues at the same rate but becomes non-productive as the newly synthesized polypeptide is specifically degraded [42]. To date, over 2000 mature human miRNAs are identified [44]. in silico prediction estimates that approximately 60% of human mRNA could be the targets of miRNA [45]. Thus, by modulating miRNA abundance and constitution, it is possible to fine tune the expression and function of proteins within the cell in a very precise manner [46]. In perspective of viral infections, modulated miRNA can impact disease progression and outcome [47, 48].

### miRNA in HBV infection

The host has a complex interaction with the virus—the host trying to suppress the virus and the virus trying to regulate the cell machinery of host for its successful proliferation. These interactions could result in either the elimination or persistence of the virus. miRNAs perform an important role in such interactions. It is notable that there is no strong proof that firmly depicts host miRNAs directly facilitates viral replication. However, there are limited evidences that show some miRNAs can enhance viral replication upon their up-regulation [49–52]. miRNAs are involved in HBV biology in multifarious ways—either viral miRNA/proteins regulating host gene expression or host miRNAs modulating viral replication and propagation [53–66]. The following Table 1 depicts the involvement of miRNAs in host viral interaction.

**Table 1:** Involvement of miRNAs in host viral interaction

	Mode of action	miRNA	Validation status	Major findings	References
miRNAs that facilitate viral replication	Host miRNA directly promote viral replication	miR-15b	Experimentally validated	Promotes HBV replication by aiding HBV enhancer I activity HNF-1α	[49]
		miR-501	Experimentally validated	Activates HBV replication by repressing HBx-interacting protein (HBXIP)	[50]
		miR-1	Experimentally validated	Enhances HBV core promoter activity by promoting farnesoid X receptor α expression	[51]
		miRs-372/373	Experimentally validated	Stimulated the production of HBV proteins and HBV core-associated DNA by targeting nuclear factor I/B	[52]
miRNAs that directly inhibit viral replication	miRNAs with target sequences in the viral genome	let-7,miR-196b, miR-433, miR-511	Computational analysis	Targets polymerase and surface genes	[53]
		miR-205	Computational analysis	Targets HBX	[53]
		miR-345	Computational analysis	Targets pre-core genes	[53]
		miR-122	Experimentally validated	Targets mRNA coding region for viral polymerase & core protein	[54]
		miR-199a-3p	Experimentally validated	Targets HBsAg coding region	[55]
		miR-210	Experimentally validated	Targets p Targets re-S1 region	[51]
		miR-125a-5p	Experimentally validated	Interacts with the HBV surface antigen	[56]
		miR-15a	Experimentally validated	Targets HBx transcript	[57]
		miR-20a, miR-92a-1, miR-16-1	Experimentally validated	Targets HBV transcripts	[58]
		miR-205	Experimentally validated	Targets HBx gene	[59]
miRNAs that indirectly inhibit viral replication	Indirectly regulates viral replication/transcription by targeting other host factors linked with viral replication	miR-122	Experimentally validated	Promotes viral replication by targeted inhibition of heme oxygenase-1	[60]
		miR-122	Experimentally validated	Targets CCNG1 and NDRG3 to inhibit viral replication	[61]
		miR-29c	Experimentally validated	Suppresses HBV replication by targeting TNFAIP3	[62]
		miR-125b	Experimentally validated	Inhibits HBV DNA intermediates and the secretion of HBsAg and HBeAg by targeted repression of SCNN1Α	[63]
		miR-141	Experimentally validated	Repress HBV replication by targeting of PPARα	[64]
		miR-155	Experimentally validated	Repress HBV replication by targeting of C/EBP-β	[65]
		miR-130a	Experimentally validated	Represses HBV replication by targeting HBV transcription enhancers PGC1α and PPAR	[66]

### miRNAs associated with different clinical stages of HBV related liver disease

A number of studies demonstrated the association of miRNA with different clinical stages of liver disease. It is worth mentioning that liver diseases with diverse clinical symptoms such as chronic liver disease (CLD), liver cirrhosis, and hepatocellular carcinoma might also occur as a consequence of multiple other infections (e.g., HCV, HDV, HAV, HEV) and exacerbating life style habit (e.g., alcohol intake, etc.) and there are miRNAs that specifically mark the clinical stage of liver disease regardless of the etiology. Those miRNAs that are particularly altered in HBV-related liver diseases has been described in Table 2.

**Table 2:** Frequently modulated miRNA expression in HBV related liver diseases

Clinical stage	miRNA	Genomic Location	Expression	Refs.
Chronic HBV	miR-122	18q21.3	Up regulation	[67, 68]
	miR- 204	9q21.12	Down regulation	[69]
	Let7c	21q21.1	Up regulation	[68]
	miR-23b	9q22.32	Up regulation	[68]
	miR-150	19 q13.33	Up regulation	[68]
Liver cirrhosis/Fibrosis	miR-29	7q32.3	Down regulation	[70–73]
	miR-133a	18q11.2	Down regulation	[74]
	miR-199	9q34.11	up regulation	[75]
	miR-214 5p	1q24.3	Up regulation	[76]
	miR-221/222	Xp11.3	Up regulation	[77]
Hepatocellular carcinoma	(*) miR-17-92 cluster	13q31.3	Up regulation	[78]
	miR-21	17q23.2	Up regulation	[78]
	miR-96	7q32.2	Up regulation	[79]
	miR-375	2q35	Up regulation	[80]
	miR-92a	5q14.3	Up regulation	[80]
	miR-101-1	1p31.3	Down regulation	[81]
	miR-199b	9q34.11	Down regulation	[81]
	miR-244	Xq28	Up regulateion	[81]
	miR-155	21q21.3	Up regulateion	[82]
	miR-122	18q21.3	Down regulation	[83]
	miR-145	5q32	Down regulation	[84]
	miR-132	17p13.3	Down regulation	[85]
	miR-34a	1p36.22	Down regulation	[58]
	miR-23a	19p13.12	Down regulation	[86]
	miR-148a	7p15.2	Down regulation	[87]
	miR-192	11q13.1	Down regulation	[88]
	miR-125b	11q24.1	Down regulation	[89]
	miR-200	1p36.33	Down regulation	[90]
	miR-602	9q34.3	Up regulation	[91]

(*) miR-17-92 cluster (miR-17, miR-18a, miR-19a, miR-20a, miR-19b-1 and miR-92a-1)

miR-122 is an established liver specific miRNA. Altered levels of this miRNA have been recorded in blood samples of HBeAg-positive chronic hepatitis patients and occult HBV infections. miR-122 is also found to be involved in neo plastic transformation and tumorigenicity, hence miR-122 abundance has been suggested as a potential HBV disease signature [67, 68]. miR-204 exhibited strong suppressive effect on HBV replication and depletion of Rab22a (target of miR-204) expression indicates antiviral effect of miR-204 [69]. miR-29 has been principally well recognized in advancement of fibrosis/cirrhosis and necro-inflammation due to its negative association with these two aforementioned clinical conditions. Fibrosis which often leads to cirrhosis primarily occurs due to collagen deposition secreted by activated hepatic stellate cells (HSCs) in the extracellular matrix of hepatocytes due to liver injury. Reports have illuminated that miR-29, through its up-regulation suppresses fibrosis/cirrhosis by repressing collagen-secreting genes in HSCs through TGF-β and NF- κB mediated pathways [70–73]. miR-133a, miR-199, miR-214 5p and miR-221/222, in contrast were found up regulated in liver fibrosis [74–77]. Association of HBV in development of HCC are hitherto documented [58, 78–91] and mainly hepatitis B virus X protein (HBx) is known to modulate a number of cellular miRNAs that facilitate the process of hepatocarcinogenesis. It is notable to mention that expression of onco-miRNAs miR-21, miR-222 and tumor suppressor miR-145 are altered differentially by the HBx protein in malignant hepatocytes [84]. A number of miRNAs can distinguish HBV related HCC from healthy controls as reported in works from Li et al. [80]. Studies have demonstrated that miR-602 increase significantly from the stage of chronic HBV infection and to reach its highest in HCC when compared with healthy liver [91].

## Exosome derived miRNAs

The pioneer study by Valadi et al. [92] that demonstrated exchange of nucleic acids through exosomes, inspected secreted exosomes from mouse and human mast cell lines. They discovered the presence of miRNAs and mRNAs of 1300 gene in exosomes which are not part of the parental cells and proposed these RNAs as exosomal shuttle RNAs (esRNAs) [92]. These esRNAs could be delivered to another cell (recipient cells), translated into functional proteins in new location [92]. This exosome mediated transport of nucleic acids discovered from this study revealed a new mechanism of cell–cell communication. This communication of genetic material between cells may be taking place in the microenvironment, but could likely occur remotely. The ability of exosomes to deliver nucleic acids in active form to cells at a distance presents a tremendous opportunity to use them as vectors for gene therapy particularly in cancer research which is discussed in the sections below.

### Secretion and uptake of exosome-derived miRNAs

The exact mechanism by which miRNA are packaged into MVBs in the endocytic pathway and secreted through exosomes is still poorly understood. However, miRNA secretion and uptake are not a random process rather a controlled one. An elaborate and extensive Study by Gibbings et al. [93] thus far have shown that MVBs are associated with GW-bodies, which are cytoplasmic foci (also coincide with P-bodies), where post-transcriptional regulation of mRNAs occurs. They are enriched in GW182 and AGO2 proteins, two main components of the RISC. Kosaka et al. have  confirmed that miRNAs are released through a ceramide-dependent secretory mechanism and a tumor-suppressive miRNA, secreted by this mechanism, was taken up by a recipient cell, where it employed gene silencing and growth inhibition [94]. As earlier mentioned, a more current study by Yeh et al. [95] has demonstrated that chronic lymphocytic leukaemia (CLL) cells secrete more exosomes in plasma than B cells from healthy donors and the exosome secretion is not spontaneous, rather their secretion is under regulation of BCR signalling pathway. Gene expression profiles and in vitro models have identified important pathways for the crosstalk between CLL cells and their microenvironment. This communication of genetic material between cells may be taking place in the microenvironment, but could likely occur remotely. The BCR is composed of membrane immunoglobulin (mIg) molecules and associated Igα/Igβ heterodimers. The mIg subunits bind with antigen causing receptor aggregation, whereas the α/β subunits transmit signals to the inside of the cell. BCR aggregation rapidly activates the Src family kinases Lyn, Blk and Fyn as well as the tyrosine kinases Syk and Btk. As a result ‘signalosome’ is formed which is composed of the BCR, the aforesaid tyrosine kinases, adaptor proteins like CD19 and BLNK, and signalling enzymes namely PLCγ2, PI3K and Vav. Signals originating from the signalosome activate multiple signalling cascades that involve kinases, GTPases, and transcription factors [96, 97]. Additionally, CLL plasma derived exosomes have unique microRNA expression compared with normal controls. miR-150 and miR-155 have significant higher expression in CLL-derived exosomes vs. normal B cells highlighting a disease-relevant exosome microRNA profile. The secretion of exosomes has been described to be controlled by increased intracellular calcium levels [98] or activation of cell surface receptors [99] or stress responses [100], suggesting that the different condition of the cell can guide the secretion and compositions of exosomes. The GW182 protein may be essential for microRNA stability and secretion through exosomes [101]. Knockdown of GW182 by siRNA enhanced microRNA instability and reduced secretion through exosomes, whereas replenishment of GW182 reinstated microRNA stability, thereby signifying a role of GW182 in protecting AGO2-bound microRNA [101].

### miRNA profiling and as cancer biomarker in Tumor-Derived exosomes

The horizontal transfer of miRNA to target cells leads to functional alterations with consequences that impact on tumor progression and metastasis [102]. A number of studies have examined the miRNA profile from circulating tumor-derived exosomes (TD-exosomes) and compared the expression levels to the original tumor cells (Fig. 1). For example, circulating TD-exosomes isolated from the serum of ovarian cancer patients and compared with, age-matched controls and primary tumor cell cultures and examined for miRNA expression. It was found that the expression of eight miRNAs, earlier established to be diagnostic in ovarian cancer, were similar between cellular and exosomal miRNAs [103]. Rabinowits et al. assessed lung adenocarcinoma patients and observed no significant differences in exosomal miRNA levels between miRNAs derived from circulating exosomes or from the primary tumors [104]. In another study, circulating exosomal microRNAs were profiled from the plasma of prostate cancer patients with and without metastases [105], and a discrete set of 11 miRNAs was documented with significantly higher level of expressions in patients having metastases than those without metastases. Overall, it was found that miRNA expression signatures are not significantly different between TD-exosomes and tumor cells [106]. With this in mind, exosome-bound miRNAs and their potential role can be utilized as genetic biomarkers of cancer. Certain number of studies, however, have shown that miRNA signatures in exosomes do not correspond to those in the parent tumor cells [107, 108]. This suggests that a sorting process occurs in the parental cell that selects and actively loads miRNAs into exosomes and that miRNA content of exosomess is specified by the type of tumor cell. Moreover, pre-miRNAs packaged into exosomes can be converted to mature mi-RNAs. Current studies have shown that breast cancer associated exosomes contain the RISC-Loading Complex which enables them to process pre-miRNAs into mature miRNAs and that the elements necessary for this maturation process, such as Dicer and CD43 are present in the exosomes [109]. Hence, TD exosomes appear as pre-programmed carriers of miRNAs, whose profile might provide important insights into the status of the parental cancer cells. Various other studies also have demonstrated that exosomes in plasma of certain cancer types, including glioblastoma [107], lung [110], breast [111] and colorectal [112] cancers, have distinct miRNA profiles. It is interesting to mention that certain miRNA species, for example miR-21, exhibited higher expression in exosomes from plasma of glioblastoma, ovarian, breast and pancreatic cancers. Also, miR-21 expression level appeared to correlate with the occurrence of disease, progression and response towards therapy [113, 114].

**Fig. 1:** microRNA profiling of circulating TD exosomes in different cancers. An overview of exosomal miRNA expression signatures in different cancers those are not significantly different between TD-exosomes and tumor cells. miRNAs marked in red color indicate miRNAs that are signature for multiple cancers, while the ones marked in blue color indicate those miRNAs that are common for 2 different cancers as depicted in Venn diagram. *TD* tumor derived

Furthermore, a database named miRandola has been developed to include all extracellular circulating miRNAs which presently contains 2312 listings with 581 unique mature miRNAs recognized in circulation from 21 different types of samples [115].

### Exosomes as a vehicle of intercellular communication

Tumor development and progression is reliant on the reciprocal relationship between cancerous cells and their neighbouring microenvironment. While the cancerous cells, that harbor many pro-tumorigenic genetic mutations, are the main driving force of tumor development, the surrounding stroma, which includes fibroblasts, endothelial and infiltrating immune cells, play a supportive and assisting role (reviewed in [116]). This relationship requires not only a particular spatial interaction, but also the ability for the cancerous cells to communicate with the adjacent microenvironment by exchanging certain soluble proteins and genetic factors. TD-exosomes are generally considered pro-tumorigenic. In the following section we will discuss about how exosomes with their cellular components makes intercellular communication between tumor cells and distant microenvironment of metastatic site, elicit pro tumorigenic effects and facilitate the pre metastatic niche formation.

#### Effects of Exosome-Derived miRNAs in pre metastatic niche formation in vivo and in patients

High recurrence and metastasis rates have become the major hindrance to improve long-term survival of HCC patients [117, 118]. Metastasis is an intricate process that comprises a series of events in which tumor cells grow, detach from the primary tumor site, invade into the circulation system and migrate to another site for tumorigenesis. The development of cancer metastases at distant organs depends on various processes like intercellular communication [119], dispersed tumor cells’ adaptation to, and co-evolution with, the radically disparate microenvironments of metastatic sites [120]. Though substantial progresses have been made in research in this field, it is unclear when and how disseminated tumor cells prime their subsequent outgrowth in the microenvironment of pre-metastatic organs.

The foundation of pre-metastatic niches, a sequence of events that prepares future metastatic sites for the inflow of tumor cells and that supports engraftment and survival of these incoming metastatic cells [121–123], has been recently shown to depend on TD exosomes [124, 125]. Tumor exosomes ‘educate’ selected host tissues towards a pro metastatic environment. Exosomes are secreted by many cells and plentifully by tumor cells [126]. Exosome binding/uptake can severely alter target cells, as demonstrated for T cell activation, immunosuppression, and conversion to a malignant phenotype [127–129].

Recent reports are emerging that exosomal miRNA from metastasizing tumor cells preferentially regulates mRNA that contributes to pre-metastatic niche formation. For e.g. matrix metalloproteinase transcription, accompanying cdh17 down-regulation, was upregulated in lymph node stroma cells (LnStr) transfected with miR-494 or miR-542-3p or co-cultured with tumor exosomes derived from metastatic rat adenocarcinoma BSp73ASML. Here tumor derived exosomes select non-transformed cells in premetastatic organs and regulate them by remote transmission of miRNA [130]. Kogure et al. showed that miRNA and protein content of exosomes derived from HCC cells differ from the cell of origin. Transforming growth factor β activated kinase-1 (TAK1) is the most likely pathway that could be modulated by these miRNAs that consequently enhance transformed cell growth in recipient cells [131]. Zhang et al. showed that both human and mouse tumor cells with normal PTEN expression, lose PTEN expression after dissemination to the brain, but not to other organs. Here brain specific astrocyte-derived exosomes facilitate an intercellular transmission of PTEN-targeting miRNAs to metastatic tumour cells. When exosome secretion from astrocyte is blocked, the PTEN activity is regained and suppresses brain metastasis in vivo [132].

Costa- Silva et al. successfully isolated pancreatic ductal adenocarcinoma (PDAC) exosomes from plasma of murine model and demonstrated sequential steps involved in the liver premetastaic niche formation mediated by PDAC derived exosomes. According to their study PDAC exosomes particularly binds with Kupffer cells of liver. They have also showed that macrophage migration inhibitory factor (MIF) was distinctly elevated in plasma exosomes of PDAC stage-1 patients who later developed liver metastasis compared to healthy controls. It suggests MIF can serve as biomarker for PDAC liver metastasis [133]. Works of You et al. revealed that Matrix metalloproteinase 13 (MMP13) was overexpressed in plasma exosomes of nasopharyngeal carcinoma (NPC) patients than healthy controls. These MMP13-containing exosomes facilitate NPC metastasis and influence tumor microenvironment causing tumor cell migration and invasion [134].

#### Pro-tumorigenic effects of exosome-derived miRNAs in vitro

Apart from regulating cell migration, inflammation, immune responses, angiogenesis, invasion, pre-metastatic niche formation- the pro-tumorigenic effects of exosome-derived miRNAs after uptake by a recipient cell have recently come to attention. Tumor-associated macrophages (TAM), which are known to stimulate invasion and metastasis, have been reported to secrete miRNA containing microvesicles that could be taken up by breast cancer cells. It was revealed that in a co-culture system, uptake of exosomes secreted from IL-4 stimulated macrophage could stimulate the invasion of breast cancer cells and interruption of the Mef2c-β-catenin pathway due to uptake of miR-223 (miRNA signature for IL-4 activated macrophages) [135]. Leukemia cell exosomes have been observed to communicate with human umbilical vein endothelial cells, culminating in increased cell migration [136]. In this study, K562 cells (leukemia cells) were transfected with a Cy3-labeled pre-miR-92a and co-cultured with HUVECs (endothelial cells). The Cy3-labeled miR-92a, derived from the K562 cells, could be identified in the cytoplasm of the endothelial cells and found co-localized with CD63 (exosome marker). Moreover, the expression of integrin α5, a target of miR-92a, was found significantly reduced in the recipient cells. This indicates that an exosome-derived miRNA can function as an endogenous miRNA in a recipient cell thereby playing a vital role in cancer-to-endothelial cell communication [136]. Process of malignant transformation may modify the pathways by which miRNAs are transported from cells, thus leading to variations in exosome content and morphology [137]. Palma et al. showed that these miRNAs are packaged and selectively exported in exosomes that are larger than conventional exosomes and are enriched in CD44 protein, a protein that is relevant to breast cancer metastasis. On the other hand, they demonstrated that normal cells release miRNAs in a homogenous type of vesicle [137].

Xiao et al. profiled the miRNAs of melanoma exosomes. They identified the 228 miRNAs that were differentially regulated in melanoma exosomes when compared with normal melanocyte exosomes, 15 of which are known to be associated with melanoma invasion and metastasis [138]. It is interesting to mention that certain secreted miRNAs may act as ligands by binding to TLRs on recipient cells. For example, miR-21 and miR-29a secreted in exosomes from lung cancer cell lines were shown to bind to murine TLR7 and human TLR8 and initiated a TLR -mediated pro-metastatic inflammatory reaction that could proceed to tumor growth and metastasis [139]. Thus it is evident from these aforementioned studies that transport of miRNAs via exosomes is indeed the machinery used by tumor exosomes as a means of intercellular communication that can begin and promote tumor advancement via transmission of genetic information at native and remote cells and tissues.

## Exosomal miRNA in liver fibrosis/cirrhosis

Cirrhosis is the end stage consequence of liver fibrosis and is strongly associated with the progression towards HCC. Liver fibrosis results from chronic liver damage in connection to inflammation and extracellular matrix (ECM) production. The predominant cell type responsible for ECM deposition is hepatic stellate cells (HSCs) and the fundamental mechanistic event of hepatic fibrosis is the activation, proliferation, and migration of HSCs. In recent times, several studies have reported on the function of exosomal miRNA in the process of liver fibrosis [140–143]. miR-214, often observed as a fibrosis associated miRNA, can likely be used as a non-invasive or minimally invasive biomarker of fibrosis progression. Connective tissue growth factor 2 (CCN2), is overexpressed in fibrotic liver and could directly promote fibrogenesis in activated HSCs [144–146]. miR-214 regulates the expression of CCN2 by directly targeting the 3′-UTR region of CCN2 and was reported to be transferred from HSCs to adjacent cells by exosomes [140]. However, miR-214 expression was decreased during chronic liver injury. Though the essential mechanism of reduced expression of exosomal miR-214 in chronic liver disease remains imprecise, isolated exosomal miR-214 or its mimic may have a therapeutic outcome on liver fibrosis. Further related and mechanistic studies will be required to explore such conflicting reports. Chen L et al., in a different study have showed that exosomal Twist1, which modulates miR-214 expression and helps CCN2 suppression in recipient cells, was down-regulated during HSC activation [141]. Repressed state of exosomal Twist1 exerts a positive influence on CCN2-dependent fibrogenesis. CCN2 could be packaged into secreted exosomes by activated HSCs and transported to other quiescent or activated HSCs [142].

## Exosomal miRNA in hepatocellular carcinoma

HCC is the primary malignancy of liver and often develops in the background of liver cirrhosis caused by its main risk factors such as HBV or HCV infection, excessive alcohol uptake etc. Obesity leading to non-alcoholic liver disease (NAFLD) and non-alcoholic steatohepatitis (NASH) is increasingly becoming one of the key etiologies for liver diseases and HCC.

Apart from the presence of mRNAs, lncRNAs and negligible amounts of ribosomal RNAs (18S and 28S rRNA), transcriptome analyses of HCC-derived exosomes revealed existence of some small RNAs in exosomes from HCC cell lines and HCC-derived primary cells compared to their parental cells e.g., HKCI-C3, HKCI-8, and MHCC97L cell lines [147, 148]. Yu et al. found that miRNAs consist of 3% of the overall small RNA population in the exosomes of HCC patient-derived cells and their lengths differ from those in the donor cells. In another study, possibly due to variations in isolation methods, miRNAs account for 2–7% of all small exosomal RNAs obtained from supernatants of HCC cells cultured in vitro [149]. Kogure et al., identified 134 miRNAs in Hep3B-derived exosomes, 11 of which (e.g., miR-584 and miR-517c) were exclusively expressed in the exosomes and not in the donor cells signifying a very high enrichment in exosomes [131].

While exosomes have been studied for quite few years, their biological importance is being recognised in cancer in recent times. The RNA and protein content in the HCC-derived exosomes differs from the exosomes derived from normal hepatocytes. Exosomes mediate inter-cellular communication, between alike as well as different cell types and most importantly exosomes from HCC or other cancers can remodel the tumor micro-environment through different methods [131]. Therefore, following section will delineate the evidences in support of the potential role of exosomal components particularly miRNAs as potential diagnostic and therapeutic biomarkers of HCC.

Wang et al. showed that exosomes derived from hepatic stellate cell can transfer miR-335-5p to the recipient HCC cells, inhibit HCC cell proliferation and invasion in vitro and can also facilitate reduction of HCC tumor in vivo [150]. Study by another group indicated that exosomal miR-21 and miR-10b induced by acidic microenvironment in HCC stimulate cancer cell proliferation and can direct the recipient cells towards a pro-metastatic phenotype [151]. In early stage HCC patients, serum exosomal miR-21 and miR-10b levels were found to be related with advanced tumor stage and HIF-1α and HIF-2α expressions [151]. These studies inform potential therapeutic strategies using miRNAs as prognostic molecular marker in HCC. Sugimachi et al. observed that exosomal miR-718 is significantly suppressed in patients with HCC recurrence after liver transplantation [152]. Decreased expression of miR-718 attributed to the poor prognosis of HCC patients by the increased expression of homeobox B8 (HOXB8). Another group obtained similar results with exosomal miR-718 for breast cancer patients [153]. Thus, exosomal miR-718 may be a novel biomarker for foreseeing HCC recurrence.

Various studies pointed towards the usefulness of miR-21 as minimally invasive potential biomarkers for early detection of HCC- whether it is HBV related or originated from some other etiological factors. Wang et al. found that exosomal miR-21 is significantly elevated in patients with HCC compared to chronic hepatitis B patients or healthy volunteers [154]. A study by Tomimaru et al. [155] showed that plasma miR-21 levels significantly reduced after curative resection in patients with HCC compared with the pre-operative values (p = 0.0125). Plasma miR-21 level in 126 patients with HCC was significantly increased than in patients with chronic hepatitis and healthy individuals (p < 0.0001, p < 0.0001, respectively). ROC analysis of plasma miR-21 yielded an AUC of 0.773 with 61.1% sensitivity and 83.3% specificity when differentiating HCC from chronic hepatitis, and an AUC of 0.953 with 87.3% sensitivity and 92.0% specificity when differentiating HCC from healthy volunteers. Both sets of values were superior to AFP and it is suggested that combination of both plasma miR-21 and AFP has a better differentiating power than plasma miR-21 and AFP alone.

Zhou et al. showed that HCC-derived exosomal miR-21 is elevated and promoted cancer progression by activating cancer-associated fibroblasts (CAFs) [156]. miR-21 converted normal HSCs to CAFs by directly targeting PTEN, led to the activation of pyruvate dehydrogenase kinase 1 (PDK1)/AKT signalling in HSCs and secreted angiogenic cytokines, including VEGF, MMP-2, MMP-9, fibroblast growth factor 2 (FGF2) and TGF β. Clinically, a high level of exosomal miR-21 correlated with CAFs, higher vessel density and survival in HCC patients. These results advocate that miR-21 may be a potential target for the treatment of HCC.

Certain exosomal miRNAs are useful in differentiating HCC from liver cirrhosis or chronic hepatitis B patients or healthy controls. Liu et al. investigated that circulating HCC patient-derived exosomal miR-125b levels were decreased compared with those from patients with chronic hepatitis B and liver cirrhosis [157]. miR-125b has been reported to be a suppressor of HCC development through the inhibition of epithelial-mesenchymal transition, tumor growth, migration, and invasion of hepatoma cells [157]. In addition, miR-125b levels in exosomes were associated with tumor number, encapsulation, and TNM stage, and showed reduced time to recurrence (TTR) and overall survival (OS). These results indicated that exosomal miR-125b could serve as a prognostic marker for HCC. Li et al. evaluated 11 familiar reference genes from circulating exosomes between healthy controls, chronic hepatitis B patients and HCC patients [158]. They observed that the combination of miR-221, miR-191, let-7a, miR-181a, and miR-26a can be an optimal gene reference set for standardizing the expression of liver-specific miRNAs for systemic analysis into the development of chronic hepatitis B to HCC [158]. Thus, exosomal miRNAs may be useful for monitoring HBV related hepatitis progression and as biomarkers to detect early stage of HBV related HCC.

## Conclusion and future direction

Several attempts have been made to investigate the propagation of chronic to advanced stage liver diseases caused by HBV. However, attempts at treatment of chronic infections or advanced liver diseases have had only limited success. Due to the exclusive dependence of HBV on the host cellular machinery [7] for its propagation and survival, investigation of the interactions between HBV and the host cell is necessary for the understanding of viral pathogenesis and development of new antiviral therapies. The discovery of miRNAs as an important modulator of gene function motivated researchers to utilize them as an expedient tool for antiviral therapy. Since then, comprehensive studies have demonstrated that many host miRNAs are modulated by the virus in order to achieve its persistence, while other miRNAs are modulated by the host with the purpose of viral clearance. Ideally circulating or exosomal miRNA may be used as biomarkers in developing minimally/non- invasive strategies for the detection of HBV-associated liver disease.

It is challenging to diagnose early-stage HCC and to treat HCC effectively. High recurrence and metastasis rates are the major obstacles to improve long-term survival of HCC patients. Surgical resection and liver transplantation are existing best curative options to treat liver cancer. However, recurrence or metastasis is fairly common in patients who have had a resection and postoperative survival rate is 30% to 70% at 5 years [reviewed in [159] ]. The foundation of pre-metastatic niches has been recently shown to depend on TD exosomes. Any biomarkers should satisfy the assay criteria not only for specificity, sensitivity, or robustness, but most importantly for clinical applicability. TD exosomes can fit the standards for a biomarker to a significant extent because they are abundant, secreted in almost all body fluids, membrane bound contents are not susceptible to degradation and imitates the parent tumor cells. They are stable and appropriately tiny to cross the blood–brain barrier. The content of TD exosomes including miRNA along with other materials allows us to analyze their molecular or genetic profiles and thereby founding tumor-specific signatures. TD exosomes have the potential of serving as a “liquid tumor biopsy” which can be obtained minimally/non-invasively and assessed frequently thereby substituting the need for a surgical or needle biopsy. During liver fibrosis, diverse exosomes are secreted to mediate fibrogenic signalling. Particular exosomes may be specific to this process and in the future they may be used as potential biomarkers for liver fibrosis. Exosomes, being a potent gene delivery system, can be the solution for the field of RNA therapeutics, whose main obstruction has been the development of a working RNA delivery system. Design of tailored synthetic exosomes during drug delivery, called “exosome mimetics” may also allow for precise targeting of cancer cells by crafting exosomes that contain cell-specific targeting molecules [132]. Even though this field is in its infancy and many hurdles will have to be overcome before exosomes will be ready for effective drug delivery system, it is reasonable to foresee all the forthcoming prospects these natural nanoparticles hold.

While the benefits offered by exosomes or specifically TD exosomes are exclusive and advantageous in many respects than that of conventional circulating cancer biomarkers, there remain several demerits with exosomes. The first and major problem is the heterogeneity of extracellular vesicle (EV)s in the body fluids of patients with cancer. Exosomes are a subcategory of EVs defined by their size, cellular origin and functional properties and TD exosomes are a further subpopulation of exosomes secreted by tumor cells. Secondly, there are no established procedures for separation of exosomes from EVs. The identity of EV populations assessed in several studies remains obscure and what is more, isolation of TD exosome is the main hurdle. As a result, in most of the cases the existing data do not differentiate TD exosomes from other EVs. Thirdly, it is still elusive which of the several exosomal constituents or signatures (such as molecular, genetic or functional) is likely to correlate better with clinical prognosis as has been reported in various studies till date.

In conclusion, many hindrances will have to be overcome before exosomes or TD exosomes with their integral signature molecules such as miRNA will be ready to function as cancer biomarkers. Nonetheless, interesting studies, especially in the field of hepato- oncology up to now and in the future may reveal that efforts necessary for further progress and substantiation of exosome-based approaches may be worthwhile.

## Data Availability

In addition to the data available in the supplementary information files, datasets used and/or analyzed during the current study are available from the corresponding author.

## Abbreviations

AFP: Alfa feto protein
BCR: Breakpoint cluster region
CAF: Cancer-associated fibroblast
CCN2: Cellular communication network factor 2
CDK: Cyclin dependent kinase
CHB: Chronic hepatitis B
CLD: Chronic liver disease
CLL: Chronic lymphocytic leukemia
CREB: cAMP response element-binding protein
CSF: Cerebrospinal fluid
DNA: De oxy ribo nucleic acid
ECM: Extracellular matrix
esRNA: Exosomal shuttle RNA (Ribo nucleic acid)
EV: Extracellular vesicle
FGF2: Fibroblast growth factor 2
GTP: Guanosine tri phosphate
HAV: Hepatitis A virus
HBcIgM: Antibody against Hepatitis B core antigen
HBeAg: Hepatitis B e antigen
HBV: Hepatitis B virus
HBsAg: Hepatitis B surface antigen
HBx: Hepatitis B virus X protein
HCC: Hepatocellular carcinoma
HCV: Hepatitis C virus
HDV: Hepatitis D virus
HEV: Hepatitis E virus
HIF-1: Hypoxia-Inducible Factor (HIF)-1
HIV: Human immunodeficiency virus
HSC: Hepatic stellate cells
Hsp: Heat shock protein
HOXB8: Homeobox B8
IL12A: Interleukin-12 subunit alpha
JAK-STAT: Janus kinase-Signal transducer and activator of transcription
LC: Liver cirrhosis
lncRNA: Long non coding RNAs
MAPK: Mitogen activated protein kinase
MAP3K: Mitogen activated protein kinase kinase kinase
MDM2: Mouse double minute 2 homologue
MIF: Migration inhibitory factor
miRNA: MicroRNA(Ribo nucleic acid)
MEF2C: Myocyte Enhancer Factor 2C
MMP: Matrix metalloproteinase
NAFLD: Non- alcoholic liver disease
NASH: Non- alcoholic steatohepatitits
NPC: Nasopharyngeal carcinoma
NPV: Negative predictive value
OS: Overall survival
PCR: Polymerase chain reaction
PDAC: Pancreatic ductal adenocarcinoma
PDC: Patient derived cells
PIK3R1: Phosphatidylinositol 3-kinase regulatory subunit alpha
PP2A: Protein phosphatase 2
PPV: Positive predictive value
PTEN: Phosphate and tensin homologue
RNA: Ribo nucleic acid
ROCK 1: Rho-associated protein kinase 1
RISC: RNA induced silencing complex
ROC: Receiver operating characteristic
RT-PCR: Real time polymerase chain reaction
SNP: Single nucleotide polymorphism
STAT: Signal transducer and activator of transcription
TAK1: Transforming growth factor β activated kinase -1
TAM: Tumor associated macrophages
TD exosome: Tumor derived exosome
TGF β: Transforming growth factor β
TLR: Toll like receptor
TTR: Time to recurrence
TNF: Tumor necrosis factor
RNA: Ribo nucleic acid
VEGF: Vascular endothelial growth factor
WHO: World Health Organization
UTR: Un-translated region
